# Neuroprotective effect of *Buyang Huanwu Decoction* on spinal ischemia-reperfusion injury in rats is linked with inhibition of cyclin-dependent kinase 5

This article has been retracted.

**DOI:** 10.1186/1472-6882-13-309

**Published:** 2013-11-09

**Authors:** Lei Wang, Dian-Ming Jiang

**Affiliations:** 1 Department of Orthopedics, First Affiliated Hospital, Chongqing Medical University, #1 Youyi Rd, Chongqing 400016, China

**Keywords:** Buyang Huanwu Decoction, Spinal ischemia-reperfusion, Cdk5, Inhibitor, Roscovitine

## Abstract

**Background:**

*Buyang Huanwu Decoction* (*BYHWD*), a traditional Chinese medicine formula, has been shown to exert a variety of pharmacological effects including neuroprotective properties. However, the mechanism of neuroprotection is not fully understood. This study was designed to explore the mechanism of *BYHWD* in the treatment of spinal ischemia-reperfusion injury in rats.

**Methods:**

Twenty-eight male Sprague–Dawley rats, weighting 250–280 g, were used, and were randomly divided into four groups with 7 animals in each: sham operation group (Control), spinal ischemia with saline (SI + Saline), spinal ischemia with *BYHWD* (SI + *BYHWD*), and spinal ischemia with roscovitine (SI + R). After 60 minutes of spinal ischemia followed by 72 hours of reperfusion, motor function of hind limbs, spinal ischemic infarction volume, the number of apoptotic cells, and cyclin-dependent kinase 5 (Cdk5) were examined.

**Result:**

Ischemia-reperfusion resulted in injury of the spines, while *BYHWD* significantly improved spinal function. The spinal infarction volume, number of apoptotic cells, and Cdk5 were decreased by administration of *BYHWD*. The similar improvements were seen with the pre-treatment of roscovitine.

**Conclusions:**

*BYHWD* prevented the ischemia-reperfusion-induced spinal injury in rats. The protective function of *BYHWD* was, in part, linked with inhibition of Cdk5.

## Background

Surgeries on the thoracic and abdominal aorta or trauma may result in paraplegia or paraphrases, as complication of spinal orthopedic procedure and thoracoabdominal aneurymectomy [1] or association of trauma [2]. Although different protective techniques have been recommended in order to lower morbidity and neurologic sequelae, using these experimental therapies as a clinical treatment is still challenging [3].

*Buyang Huanwu Decoction* (*BYHWD*), a well-known traditional Chinese medicine formula, has been used for the treatment of paralysis and stroke for hundreds of years, and has increasingly gained attention due to its significant neuroprotective properties. Clinical efficacy of *BYHWD* in the neuroprotective effects has been reported recently [4]. The reported mechanisms of *BYHWD* on the treatment of ischemic brain and spinal injuries have involved the thioredoxin system [5] and glutamate [6]. Those published findings, however, cannot fully explain the neuroprotective mechanisms of *BYHWD* on spinal ischemia-reperfusion injury, and other different factors may be involved in the protective mechanisms.

Cyclin-dependent kinase 5 (Cdk5) has been shown to be crucial for neuronal migration in the spinal cord [7,8], and to exert beneficial effects on the ischemia-reperfusion injury in the neuronal system [9]. The expression of Cdk5 is up-regulated during neuronal death in response to different toxic stimuli [10,11]. Thus, reducing activation of Cdk5 seems to be very important in the treatment of spinal ischemia-reperfusion injury.

We have speculated that the therapeutic effect of *BYHWD* on spinal ischemia-reperfusion injury may link with the reduction of Cdk5. Therefore, the present study was designed to explore if Cdk5 was involved in the underlying therapeutic mechanism of *BYHWD*.

## Methods

All animal care complied with the guidelines for laboratory animals, and the study was approved by the Ethics Committee of Chongqing University.

### Composition and preparation of BYHWD

*BYHWD* is composed of *Radix Astragali* (120 g), *Radix Angelicae Sinensis* (6 g), *Radix Paeoniae Rubra* (6 g), *Rhizoma Chuanxiong* (3 g), *Semen Persicae* (3 g), *Flos Carthami* (3 g) and *Lumbricus* (3 g). All dried crude drugs were provided by Jiangsu Pharmacy Company (Nanjing, China), identified by the Department of Pharmacology, Chongqing Medical University, and mixed in the ratio of 120:6:6:3:13:3:3. The herbs were decocted by boiling in distilled water for 30 minutes. The solution was then freeze-dried under vacuum, and made into a powder. The powder was dissolved in distilled water to a final concentration of 5 g/ml (equivalent to dry weight of raw materials).

### Experimental Animals and Induction of Spinal Cord Ischemia-reperfusion

Twenty-eight male Sprague–Dawley rats, weighting 250–280 g, were used in the study. The animals were randomly divided into four groups with 7 animals in each: sham operation group (Control), spinal ischemia with saline (SI + Saline), spinal ischemia with *BYHWD* (SI + *BYHWD*), and spinal ischemia with roscovitine (SI + R).

Spinal cord ischemia-reperfusion was induced by using the previously described method [5]. All animals were anesthetized with chloral hydrate (350 mg/kg) administered intraperitoneally. The temperature was continuously monitored with a rectal probe inserted 5 cm into the rectum. The temperature was maintained at 37 ± 0.5°C with an infrared heat lamp and a heating pad. The femoral artery was cannulated with a polyethylene tube (PE-50) to facilitate continuous monitoring of heart rate and arterial blood pressure, and for collecting blood samples for the analysis of blood gases and blood pH. Laser-Doppler flowmetry was recorded continuously during surgery using a method described previously [5]. Ischemia of the lumbar spinal cord was produced by occlusion of the abdominal aorta 0.5 cm below the left renal artery for 60 minutes, followed by 72 hours of reperfusion. Sham operation rats underwent the same procedure, but no occlusion of the aorta was performed.

Rats in the both SI + Saline and SI + *BYHWD* groups were administered with 8 ml of saline and 40 g/kg of *BYHWD*, respectively, by intragastric infusion, starting at reperfusion, 30, 60, 120, 240 and 360 minutes after reperfusion, and then the same dose was infused every 24 hours for 3 days. The dosage of *BYHWD* was chosen as previously described [5].

To examine whether Cdk5 was involved in apoptosis caused by spinal ischemia-reperfusion*,* the selective inhibitor of Cdk5, roscovitine, was used in the SI + R group. Roscovitine was dissolved in dimethyl sulfoxide following the previously reported method [8]. 30 mg/kg roscovitine in a volume of 8 ml was intravenously administrated 30 min before spinal ischemia started.

### Examination of motor function

After 72 hours of reperfusion, twenty-eight Sprague–Dawley rats were evaluated for the motor function of the hind limbs using Tarlov Scoring System [12]. The system was used to score neurological function as follows: 0, complete flexion; 1, severe incomplete flexion; 2, could move, but could not jump; 3, jump with obvious instability; 4, jump with slight instability; and 5, normal motor function.

### Examination of spinal ischemic infarction volume

After examination of motor function following 72 hours of reperfusion, rats were sacrificed under deep isoflurane anesthesia, quickly removed the spines, and measured the infarct volume of spines. 2-mm sections were made, stained with 2% triphenyltetra zolium chloride, and fixed in PBS. The infarction volume was determined by using the ImageJ software (National Institutes of Health, U.S.).

### Examination of apoptosis quantity

After the evaluation of the motor function and infarction volume, the L_2-3_ of lumbar spinal cord was taken. Terminal deoxynucleotidyl transferase dUTP nick end labeling (TUNEL) technique was performed using an in situ apoptosis detection kit (Intergen Company, USA.). The total number of TUNEL-positive cells on each section was counted, and expressed as the TUNEL index.

### Examination of Cdk5, p35 and p25

Following 72 hours of spinal ischemia-infusion, all animals were scarified, spinal cord was quickly removed. The lumbar spinal cords were homogenized on ice in lysis buffer. For analysis of p35/p25 protein expression, the protein extracts were electrophoresed on a 12% acrylamide SDS polyacrylamide gel electrophoresis and immunoblotted onto polyvinylidene fluoride membranes. The membranes were incubated with primary antibodies against p35/p25 (Cell Signaling Technology, Beverly, MA, USA), and blocked for 1 hour at room temperature, or primary antibodies against β-actin as an internal control dilution. The bands were visualized by ECL Western blotting analysis system (Amersham Pharmacia Biotech Europe, Freiburg, Germany). Band intensity was quantified by using an image analyzer (Raytest Isotopenmessgeräte, Straubenhardt, Germany). For analysis of Cdk5 level and activity, Western blot and immunoprecipitation kinase activity assays were respectively performed as previously described [13,14]. Cdk5 activity was expressed as an integrated optical density.

### Statistical study

Data were expressed as mean ± SEM. Statistical analysis of the neurologic scores was analyzed by Mann–Whitney non-parametric test. Differences for each Cdk5 level were analyzed by one-way ANOVA for multiple comparison tests across time points with SPSS11.0 software. A P value less than 0.05 were considered to be statistically significant.

## Results

Before, during and after the procedure, heart rate, blood pressure, and body temperature were kept within normal ranges, and were similar in all groups. All animals completed the study.

### Administration of BYHWD and pre-treatment of roscovitine improved the motor function

Spinal ischemia for 60 minutes, followed by 72 hours of reperfusion, resulted in a significant motor function deficit, but administration of *BYHWD* greatly improved the function (P < 0.05). The pre-administration of roscovitine significantly improved the function (P < 0.05). There was no significant difference between *BYHWD* and roscovitine groups, even if the Scoring index was higher in roscovitine group than that in *BYHWD* group (Figure 1).

**Figure 1:** **The motor function evaluated by Tarlov Scoring System after 72-hour reperfusion.** The spinal ischemia-reperfusion significantly impacted the motor function, and a high score was seen in animals with spinal ischemia + saline; but *BYHWD* administration and roscovitine pre-treatment greatly improved the motor function. The score was higher in the group with roscovitine than that in the group with *BYHWD*, but there were no significant differences between the groups. **: P < 0.01 *vs.* Control group. *#: P < 0.05 *vs.* SI + Saline. SI + Saline: Spinal ischemia + Saline. SI + *BYHWD*: Spinal ischemia + *BYHWD.* SI + R: Spinal ischemia + Roscovitine.

### Administration of BYHWD and pre-treatment of roscovitine reduced the spinal ischemic infarction volume

Spinal ischemia for 60 minutes, followed by 72 hours of reperfusion, resulted in an extensive spinal infarction volume, while administration of *BYHWD* greatly reduced the infarction volume (P < 0.05). The pre-administration of roscovitine also significantly reduced the infarction volume (P < 0.05). There was no significant difference between *BYHWD* and roscovitine groups, even if the infarction volume was higher in roscovitine group than that in *BYHWD* group (Figure 2).

**Figure 2:** **The volume of spinal infarct 72 hours after reperfusion.** A great infarction volume was seen in the ischemic group, but infarction volumes were largely decreased in the animals with *BYHWD* administration, and roscovitine pre-treatment. The infarction volume was lower in the group with *BYHWD* than that in the group with roscovitine; but there was no significant difference between the two groups. **: P < 0.01 *vs.* Control group. *#: P < 0.05 *vs.* SI + Saline. SI + Saline: Spinal ischemia + Saline. SI + *BYHWD*: Spinal ischemia + *BYHWD.* SI + R: Spinal ischemia + Roscovitine.

No TUNEL-positive cells were seen on sham-operated sections, but a large number of apoptotic cells was observed on the ischemic tissues of the saline group. The number of TUNEL-positive cells was significantly lower in the *BYHWD* group than in the saline group (P < 0.01). The administration of roscovitine decreased the number of TUNEL-positive cells, but the number was higher than that in the *BYHWD* group, although there was no significant difference between the two groups (Table 1).

**Table 1:** TUNEL indices in the spinal cord after spinal ischemia/reperfusion

**Group**	**Apoptosis Index (%)**
*BYHWD*	7.92 ± 2.1^a^
Roscovitine	7.01 ± 1.2^a/c^
Saline	12.39 ± 2.7^b^
Sham	0.03 ± 0.01

^a^: P < 0.01, compared to the saline group.

^b^: P < 0.01, compared to the sham group.

^c^: No significant difference, compared to *BYHWD* group.

*BYHWD* group: spinal ischemia/reperfusion group with *BYHWD* infusion.

Roscovitine group: spinal ischemia/reperfusion group with pretreatment of roscovitine.

Sham group: sham-operated group.

Saline group: spinal ischemia/reperfusion group with saline infusion.

*BYHWD*: Buyang Huanwu Decoction.

#### Alteration of p35 and p25 expressions after spinal ischemia-reperfusion

The expressions of both p35 and p25 were changed by ischemia-reperfusion: p35 was significantly down-regulated, while p25 was up-regulated after ischemia-reperfusion, suggesting that p25 was up-regulated via an elevation of cleavage of p35 (Figure 3). Alteration of p35 and p25 resulted in a hyper-activation of Cdk5.

**Figure 3:** **Expressions of p35 and p25 were alternated after spinal ischemia-reperfusion injury.** p25 was up-regulated **(A)**, p35 was down-regulated **(B)**, and Western blot was performed for analysis of expressions of p35 and p25 **(C)** after spinal ischemia-reperfusion injury. Administration of *BYHWD* and roscovitine influenced the alteration of both p25 and p35 expressions. *: *P* < 0.05, SI + *BYHWD vs.* SI + Saline group. *: *P* < 0.05, SI + R *vs.* SI + Saline group. ** *P* < 0.01, SI + Saline *vs.* Control group. SI + Saline: Spinal ischemia + saline. SI + *BYHWD*: Spinal ischemia + *BYHWD.* SI + R: Spinal ischemia + Roscovitine.

### Elevation of Cdk5 activity and level after spinal ischemia-reperfusion

Activity and level of Cdk5 were significantly elevated after spinal ischemia-reperfusion injury. Administration of roscovitine greatly inhibited Cdk5. The decrease in Cdk5 activity and level was also seen by the administration of *BYHWD*, indicating that *BYHWD* protected spine from ischemia-reperfusion injury through inhibition of Cdk5 (Figure 4).

**Figure 4:** **Cdk5 activity and level after spinal ischemia-reperfusion injury.** Cdk5 activity was significantly elevated after spinal ischemia-reperfusion injury. The administration of *BYHWD* and roscovitine greatly inhibited Cdk5 activity **(A)**. The similar results were confirmed in Western blot, showing that spinal ischemia-reperfusion resulted in an elevation of Cdk5 level, and that *BYHWD* and roscovitine inhibited Cdk5 level **(B)**. β-Actin was used as a loading control. *#: *P* < 0.05, *vs.* SI + Saline group. ** *P* < 0.01, *vs.* Control group SI + Saline: Spinal ischemia + saline. SI + *BYHWD*: Spinal ischemia + *BYHWD*. SI + R: Spinal ischemia + Roscovitine.

## Discussion

In clinical practice, acute spinal ischemia may result in a major clinical disability due to spinal infarction. For several centuries, *BYHWD* has been used as a traditional medicine for the treatment of cerobrovascular and spinal diseases in eastern medicine. Some available studies on spinal injury have been reported [15,16], but further exploration of the exact mechanisms of *BYHWD* in the neuroprotective therapy is needed. Different factors including oxidative stress [17] and excitotoxic stimulation [18], which are involved in neuronal apoptosis, have been reported. A most recent study demonstrated that the neuroprotective therapy of *BYHWD* for spinal ischemia-reperfusion injury was through a decrease in apoptosis [5]. The present study, using animal model, confirmed that *BYHWD* prevented the ischemia/reperfusion-induced spinal injury, and demonstrated that the protective function of *BYHWD* was, in part, through the inhibition of Cdk5.

Apoptosis is an important mechanism in the pathogenesis of the secondary injury process following spinal cord injury [19]. Apoptosis is an active gene-directed death process mediated by activation of a number of cysteine proteases; therefore, it may be preventable with selective inhibitors. Cdk5 is a member of the Cdk family of serine/threonine kinases [18], and is crucial for neuronal migration in the spinal cord [7,8]. Cdk5 activity is triggered by its activator p35 [20]. Under pathological conditions, p35 is cleaved into a shorter form p25. The p25 fragment triggers Cdk5 hyper-activation and translocation of the p25/Cdk5 complex to the cytoplasm where it hyper-phosphorylates a number of substrates, leading to neuronal death [21]. Roscovitine is a potent selective inhibitor of Cdk5, and exerts protection from ischemia-reperfusion injury in the neuronal system [9]. Many evidences have demonstrated that administration of roscovitine inhibits Cdk5 activity, and prevents neuronal apoptosis.

The present study showed that ischemia-reperfusion injury caused alterations of p25/p35, specifically in up-regulated expression of p25 and down-regulated expression of p35. These findings suggested that spinal ischemia-reperfusion triggered the activation of Cdk5 through cleavage of p35 to p25. Activation of Cdk5 results in neuronal apoptosis, inhibition of Cdk5 protects neurons from apoptosis [22]. Cdk5 inhibitor inhibits activity of Cdk5 [23], and reduces neuronal apoptosis or cell death [23,24]. In this study, the selective inhibitor of Cdk5, roscovitine, was administrated before spinal ischemia-reperfusion injury was made. The results from the present study demonstrated that apoptosis was greatly prevented, and motor function was significantly improved. Thus, these findings suggested that the neuronal apoptosis was linked with activation of Cdk5, and that Cdk5 inhibitor, roscovitine, prevented the apoptosis, and improved the motor function. These could explain the protective mechanisms of *BYHWD* therapy, because the similar protective outcome was demonstrated in the animals administrated with *BYHWD*. Therefore, the roscovitine-like protection of *BYHWD* strongly suggested that the therapeutic mechanism of *BYHWD* for the spinal ischemia-reperfusion injury was linked with reduction of Cdk5.

Moreover, the neuroprotections of *BYHWD* against the cellular apoptosis, motor function, and spinal infarction caused by spinal ischemia-reperfusion injury could be due to the fact that *BYHWD* not only inhibited Cdk5, but also influenced other previously reported factors including oxidative stress [7], glutamate [8], DNA damage and thioredoxin system [5]. Roscovitine selectively inhibited Cdk5 only, while *BYHWD* influenced multiple factors. Therefore, findings from the present study were of importance for the further exploration of multiple mechanisms in respond to the spinal ischemia-reperfusion injury.

## Conclusions

Spinal ischemia-reperfusion caused a number of spinal neuronal apoptosis and significantly damaged motor function, while administration of *BYHWD* greatly prevented those injuries. Inhibition of Cdk5 activity by roscovitine evidently protected the neuronal cells against apoptosis or death. Our results in the present study suggested that hyperactivity of Cdk5 was involved in the pathogenesis of ischemia/reperfusion-induced spinal neuron apoptosis, and that *BYHWD* protected the spine against ischemia-reperfusion injury partly through the inhibition of Cdk5.

## Abbreviations

BYHWD: Buyang Huanwu Decoction; Cdk5: Cyclin-dependent Kinase 5; SI: Spinal Ischemia; R: Roscovitine; TUNEL: Terminal deoxynucleotidyl transferase dUTP nick end labeling.

## Competing interests

The authors declare that they have no competing interests.

## Authors’ contributions

LW carried out the molecular genetic studies, participated in the sequence alignment and drafted the manuscript. DMJ participated in the design of the study and performed the statistical analysis. Both authors read and approved the final manuscript.

## Pre-publication history

The pre-publication history for this paper can be accessed here:

http://www.biomedcentral.com/1472-6882/13/309/prepub
